This article has been retracted.

# Rocaglamide Prolonged Allograft Survival by Inhibiting Differentiation of Th1/Th17 Cells in Cardiac Transplantation

**DOI:** 10.1155/2022/2048095

**Published:** 2022-01-17

**Authors:** Chen Dai, Xi Zhou, Lu Wang, Rumeng Tan, Wei Wang, Bo Yang, Yucong Zhang, Huibo Shi, Dong Chen, Lai Wei, Zhishui Chen

**Affiliations:** ^1^Institute of Organ Transplantation, Tongji Hospital, Tongji Medical College, Huazhong University of Science and Technology; Key Laboratory of Organ Transplantation, Ministry of Education; NHC Key Laboratory of Organ Transplantation; Key Laboratory of Organ Transplantation, Chinese Academy of Medical Sciences, Wuhan, China 430030; ^2^Department of Immunology, School of Basic Medicine, Tongji Medical College, Huazhong University of Science and Technology, Wuhan, China 430030; ^3^Department of Geriatrics, Tongji Hospital, Tongji Medical College, Huazhong University of Science and Technology, Wuhan, China 430030

## Abstract

**Background:**

Aglaia (Meliaceae) species are used for treating autoimmune disorders and allergic diseases in Asian countries. Rocaglamide, an extract obtained from Aglaia species, exhibits suppressive effect by regulating the T cell subset balance and cytokine network in cancer. However, whether it can be used in organ transplantation is unknown. In this study, we investigated the antirejection effect and mechanism of action of rocaglamide in a mouse cardiac allograft model.

**Methods:**

Survival studies were performed by administering mice with phosphate-buffered saline (PBS) (*n* = 6) and rocaglamide (*n* = 8). Heart grafts were monitored until they stopped beating. After grafting, the mice were sacrificed on day 7 for histological, mixed lymphocyte reaction (MLR), enzyme-linked immunosorbent assay (ELISA), and flow cytometric analyses.

**Results:**

Rocaglamide administration significantly prolonged the median survival of the grafts from 7 to 25 days compared with PBS treatment (*P* < 0.001). On posttransplantation day 7, the rocaglamide-treated group showed a significant decrease in the percentage of Th1 cells (7.9 ± 0.9% vs. 1.58 ± 0.5%, *P* < 0.001) in the lymph nodes and spleen (8.0 ± 2.5% vs. 2.4 ± 1.3%, *P* < 0.05). Rocaglamide treatment also significantly inhibited the production of Th17 cells (6.4 ± 1.0% vs. 1.8 ± 0.4%, *P* < 0.01) in the lymph nodes and spleen (5.9 ± 0.3% vs. 2.9 ± 0.8%, *P* < 0.01). Furthermore, the prolonged survival of the grafts was associated with a significant decrease in IFN-*γ* and IL-17 levels. Our results also showed that NF-AT activation was inhibited by rocaglamide, which also induced p38 and Jun N-terminal kinase (JNK) phosphorylation in Jurkat T cells. Furthermore, by using inhibitors that suppressed p38 and JNK phosphorylation, rocaglamide-mediated reduction in NF-AT protein levels was prevented.

**Conclusion:**

We identified a new immunoregulatory property of rocaglamide, wherein it was found to regulate oxidative stress response and reduce inflammatory cell infiltration and organ injury, which have been associated with the inhibition of NF-AT activation in T cells.

## 1. Introduction

Organ transplantation is an effective therapy for patients with end-stage organ disease [1]. The oxidative stress caused by the infiltration of inflammatory cells in cardiac allografts results in the production of cytokines and proinflammatory adhesion molecules, which are the main alloantigen-independent factors leading to allograft vasculopathy and organ injury [2]. Previous studies have focused on developing the optimum function of allografts by using immunosuppressive drugs, which are important for investigating the precise cell-mediated immune response and finding a way to downregulate the specific immunoreaction. Eventually, these drugs can reduce the secretion and chemotaxis of inflammatory factors and reduce oxidative stress damage and protect the allograft.

The differentiation of CD4+ T cells is induced by helper T cells, including Th1, Th17, Th2, and regulatory T cells (Tregs). Th1 cells play a key role in triggering immunoreaction, promoting inflammatory infiltration, and exacerbating oxidative stress, and several studies have shown that these types of cells increase the risk of allograft injury and allograft rejection [3, 4].

Naïve CD4+ T cells are usually activated and induced to differentiate into Th1 and Th17 cells, especially in an inflammatory environment. Interleukin-2 (IL-2) and interferon-*γ* (IFN-*γ*) secreted by Th1 cells can upregulate the production of cytotoxic T lymphocytes, elicit an immune response, and stimulate the activation of natural killer cells. Several studies have shown that Th17 cells are involved in triggering various immune processes such as Th1 cell-mediated inflammation, disordered oxidative stress, and tissue damage after organ transplantation [5]. Interleukin-17 (IL-17) secreted by Th17 cells can induce the production of many cytokines, thus increasing the count of neutrophilic granulocytes and promoting the migration of macrophages to the allograft site. Furthermore, allografts exhibit upregulated levels of IFN-*γ* and IL-17 in the serum in case of acute rejection, which is dangerous and causes inflammatory diseases compared with those with a functional and effective allograft in a transplant model [6]. Acute rejection is observed within 7 days after transplantation in the transplantation models, characterized by binding of different cellular immunoreaction and inflammatory factors, as well as natural antibodies and the oxidation-related epitope malondialdehyde. This rejection results in vascular endothelial damage, vasculitis, thrombosis, tissue destruction, and edema [7–9]. Memory T cells are also an obstacle for transplantation because 40–50% of T cells circulating in the peripheral blood have memory phenotypes [10].

Rocaglamide has attracted attention as a new anticancer drug because it can block the nuclear factor-*κ*B (NF-*κ*B) pathway [11, 12] and can also be used to treat allergic inflammatory and skin diseases [13]. Recently, rocaglamide derivatives have been demonstrated the negatively regulated effects of T cells [12, 14]. Some studies have shown that these derivatives play a crucial role in inhibiting the phorbol myristate acetate- (PMA-) induced expression of NF-*κ*B target genes and sensitizing leukemic T cells to apoptosis induced by tumor necrosis factor-*α* (TNF-*α*) [12]. Interestingly, rocaglamide suppresses the expression of tumor-related cytokines in the peripheral blood [12, 15]. Several inducible transcription factors, including NF-*κ*B and nuclear factor-AT (NF-AT), can regulate the expression of IL-4, IFN-*γ*, and TNF-*α* [16, 17]. Ca2+-dependent phosphatase calcineurin is activated after the activation of T cells, and thus, these reactions promote the dephosphorylation of NF-AT and their transfer to the nucleus [18]. In the nucleus, a representative productive immunoreaction is induced by the NF-AT protein that synergizes with activator protein 1 (AP1) and other transcription factors. Interestingly, the impairment of NFAT1 and NFAT2 in T cells is related to the severe reduction in the levels of many cytokines such as IFN-*γ*, interleukin-4 (IL-4), interleukin-10 (IL-10), colony-stimulating factor, and TNF. A previous study has shown that the TH1/TH2 lineage selection is decided by the NF-AT protein in cooperation with signal transducer and activator of transcription factors, such as STAT4 downstream of IFN-*γ* for TH1 cells and STAT6 downstream of IL-4 for TH2 cells [19]. Accordingly, the dephosphorylation and transfer of the NF-AT protein lead to the activation and differentiation of T cells, promoting secretion, chemotaxis, and adhesion of corresponding inflammatory factors and exacerbating the injury of oxidative stress and dysfunction of the allograft.

Therefore, we hypothesized that rocaglamide could be used for cell-mediated acute rejection for preventing helper T cell differentiation and T cell-mediated cytokine secretion. To confirm this hypothesis, we developed the mouse allo-cardiac transplantation model, where the donor's heart was transplanted to the abdominal vessels of the recipient. We then studied the effect of rocaglamide treatment on the immune response elicited by the infiltration of inflammatory cells and the induction of oxidative stress.

We found that rocaglamide is a potent immunosuppressive agent that can inhibit T cell proliferation and reduce the infiltration of inflammatory cells. We also found that it can downregulate the Th1 response and decrease the number of Th1 and Th17 cells in the spleen and lymph nodes. Furthermore, rocaglamide inhibited the activity of NF-AT; however, there was no inhibitory effect on the NF-*κ*B activity when rocaglamide was used at a concentration of 100 nM. On the other hand, the reduction in IFN-*γ* and IL-17 levels could be detected in the peripheral blood.

## 2. Materials and Methods

### 2.1. Animals

Female C57BL/6 (B6, H-2b) and BALB/c (H-2d) mice (age: 8–12 weeks) were purchased from Vital River Laboratory Animal Technology Co., Ltd., Beijing, China. All animals were bred in a specific pathogen-free facility of the Key Lab of Organ Transplantation Institute with (22°C, 50% air humidity, and air change). Unlimited access to food and water was provided. Mice (weighing: 22–28 g) were used as donor and recipient, respectively. All procedures were approved by the guidelines of the Institutional Animal Care and Use Committee (IACUC).

### 2.2. Heart Transplantation Model

The hearts from BALB/c were transplanted into the abdominal vessels of C57BL/6 recipients using the microsurgical technique of Luan et al. [20]. Graft survival was monitored daily by palpation. Rejection was defined as the complete loss of a palpable heartbeat [21].

### 2.3. Drug Treatment

Rocaglamide (>98% pure) was procured from ChromaBio (Chengdu, China). The recipients were treated with rocaglamide for 2 weeks (2.5 *μ*g/g in 50 *μ*l phosphate-buffered saline (PBS); intraperitoneal injection (ip); *n* = 8), and the others received PBS alone as control [22].

### 2.4. Cells and Cell Culture

RPMI-1640 medium supplemented with 10% fetal bovine serum (FBS) was used to maintain the Jurkat T leukemia cells (acquired from Clontech) under a 5% CO_2_ atmosphere at 37°C [23].

### 2.5. Histological Analysis

The grafts were resected from the recipient mice on day 7 after transplantation and analyzed by light microscopy. The specimens were fixed with 10% phosphate-buffered formalin, embedded in paraffin, and sliced into 5 *μ*m thick sections. After staining with hematoxylin and eosin (H&E), the samples were analyzed in a blinded manner. According to the International Society of Heart and Lung Transplantation (ISHLT) standard, classification was performed based on the degree of infiltration and the distribution location of inflammatory cells in the grafts [21, 24].

### 2.6. Mixed Lymphocyte Reactions (MLR)

T lymphocytes isolated from the recipient's spleens using nylon wool columns (Wako, Osaka, Japan) were used as responder cells, while donor mouse spleen cells were used as stimulator cells. The responder cells (5 × 105 cells) were cocultured with the stimulator cells (5 × 104 cells), which were then treated with mitomycin (40 *μ*g/ml, Amresco, Solon, OH, USA) in 200 *μ*l of RPMI 1640 supplemented with 10% FBS and 1% penicillin and 1% streptomycin. Then, the cells were cultured at 37°C under a humidified atmosphere with 5% CO_2_ for 3 days. The proliferation of the T cells was detected by using the BrdU enzyme-linked immunosorbent assay (ELISA) Kit (MultiSciences, Hangzhou, China). The optical density (OD) values were quantified by an ELISA reader (Model 680, Bio-Rad, Hercules, California, USA).

### 2.7. ELISA

Peripheral blood was gathered via cardiac puncture. The expression of IFN-*γ*, IL-6, and IL-17 were determined by using a commercial ELISA kit (MultiSciences, Hangzhou, China) in the culture supernatants and peripheral blood samples.

### 2.8. Flow Cytometry

The recipients were sacrificed on day 7 for the test experiments. T lymphocytes from the lymph nodes of the recipient mice (1 × 106 cells/100 *μ*l) were stained using fluorochrome-labeled antibodies in accordance with the manufacturer's instructions. Antibodies used for flow cytometric analysis were IFN-*γ*, IL-17, and CD4 (all from eBioscience). The objective cells harvested per tube ranged from approximately 15000 to 20000, of which 2000 cells were analyzed inside the lymphocyte gate. The stained cells were performed using the Becton-Dickinson FACSCalibur™ System; BD Biosciences, Franklin Lakes, NJ, USA, and analyzed using the FlowJo software (Tree Star Inc., Ashland, OR).

### 2.9. Western Blotting

Jurkat T cells were stimulated with PMA and ionomycin for 2 h with or without rocaglamides, which were added an hour before stimulation. Nuclear proteins were separated and immunoblotted with the antibody against NFATc1. The widely used p38 kinase and Jun N-terminal kinase (JNK) inhibitors, SB203580 and SP600125, were purchased from Selleck. Western blotting was performed, as described previously [12, 25]. Anti-NF-ATc1 mAb (7A6; Alexis Biochemicals) was used for detection purposes.

### 2.10. Quantitative Real-Time PCR (qRT-PCR)

According to the instruction of manufacturer, RNA was extracted from the grafts of recipient mice using TRIzol Reagent (Invitrogen, Carlsbad, CA). The primer sequences used are as follows: IFN-*γ* (forward 5′-CGGCACAGTCATTGAAAGCCTA-3′, reverse 5′-GTTGCTCATGGCCTGATTGTC-3′), IL-10 (forward 5′-GACCAGCTGGACAACATACTGCTAA-3′, reverse 5′-GATAAGGCTTGGCAACCCAAGTAA-3′), and transforming growth factor beta (TGF-*β*) (forward 5′-TGACGTCACTGGAGTTGTACGG-3′, reverse 5′-GGTTCATGTCATGGATGGTGC-3′). Each gene expression was normalized with GAPDH mRNA content: R-*β*-actin (forward 5′-CATCCGTAAAGACCTCTATGCCAAC-3′, reverse 5′-ATGGAGCCACCGATCCACA-3′) and ROR-*γ*t (forward 5′-GCTCCCGGCCTGGTCTGCTC-3′, reverse 5′-AGGTGGCGGGGTGGTTTCTGA-3′).

### 2.11. Statistical Analyses

Specimens were analyzed in duplicate or triplicate, and the data were presented as the mean ± standard deviation from one representative experiment of at least three experiments. The mean survival time of each group was determined using the Kaplan-Meier method and log-rank test. Data of statistical significance were analyzed using a *t*-test. *P* < 0.05 was considered to be a statistically significant; *P* < 0.01 and *P* < 0.001 indicated highly significant differences. All analyses were performed using the GraphPad Prism 5.0 software (GraphPad Software, Inc., San Diego, CA).

## 3. Results

### 3.1. Administration of Rocaglamide Further Prolongs Graft Survival

First, we performed heterotopic cardiac transplantation. Recipients were treated with rocaglamide (2.5 *μ*g/g in 50 *μ*l PBS; ip; *n* = 8), and the control group was treated with PBS (50 *μ*l PBS; ip; *n* = 6). The median survival of grafts (time for rejection) in the rocaglamide-treated group was 25 days compared to that in the control group (7 days; *P* < 0.001). We then determined the effect of rocaglamide on allograft survival. Grafts harvested from B6 recipients of the rocaglamide-treated group showed significantly reduced inflammatory cell infiltration and relatively normal myocardial area on day 7 than that in the control group, in which we found considerable inflammatory cell infiltration and morphological damage (Figures 1(a) and 1(b)).

We analyzed the ISHLT scores of the hearts (Figure 1(c)). Allografts from the control group showed pathological changes such as edema and congestion in myocardial tissues (scores ranged from 3 to 4). However, the rocaglamide-treated group showed normal histological characteristics, with scores ranging between 1 and 2. These findings revealed that rocaglamide inhibited the infiltration of inflammatory cells, such as neutrophilic granulocytes, and also prevented their migration.

### 3.2. Administration of Rocaglamide Inhibits the T Cell Activation in Allograft Recipients

Freshly isolated lymphocytes and splenocytes were stained for determining CD3, CD134 (OX40), CD69, and CD44 expression and assayed for detecting T cell activation in the transplantation recipients. As shown in Figure 2(a), compared with the number of CD3+ cells in the control group (5.88%), that in the rocaglamide-treated recipients (19.6%) was suppressed significantly in the lymph nodes and spleen (29.4% vs. 18.8%; *P* < 0.05). To understand how rocaglamide treatment affected T cell activation, the levels of CD134, CD69, and CD44 were determined. We found that the levels of CD134 and CD69, considered as indicators of T cell activation, decreased in the lymph nodes and spleen of the treatment group than in the control group (Figures 2(f) and 2(g)). However, there was no significant difference in the level of CD44 (Figure 2(h)). Therefore, these findings indicate that during immune activation, rocaglamide could have suppressed the proliferation of T lymphocytes by inhibiting the levels of CD134 and CD69.

We also found that in the case of CD11b+ and CD11c+ antigen-presenting cells in the spleen, rocaglamide caused a slight increase in the number of CD11b+ cells (Figure 2(b)), but this increase was not statistically significant, and rocaglamide treatment had no difference in the number of CD11c+ cells (Figure 2(c)). Furthermore, a slight increase in the number of CD11b+ CD80+ cells was observed more in the spleen of the treatment group than that of the control group (8.77% vs. 12.3%, Figure 2(d)); however, there was no difference in the number of CD11c+ CD86+ cells (Figure 2(e)). These effects may have been caused by the inhibition of T cell activation by rocaglamide, resulting in the ineffective proliferation of antigen-presenting cells.

### 3.3. Rocaglamide Administration Decreases the Number of Th1 Cells, Cytokine Expression by Th1 T Cells, and Accumulation of IFN-*γ* in Allograft Recipients

To evaluate the effect of rocaglamide treatment on the number of Th1 cells, which differentiate from CD4+ T cells in an inflammatory environment, lymphocytes and splenocytes were isolated and stained with fluorochrome-conjugated-specific antibodies and analyzed by flow cytometry. We found that the number of CD4+ IFN-*γ*+ (Th1) cells in the rocaglamide-treated group was markedly suppressed. The percentage of Th1 cells in lymph nodes of the treatment group decreased to 1.33% compared with that in the control group (7.67%; *P* < 0.001; Figure 3(a)). Furthermore, the same decrease in CD4+ IFN-*γ*+ (Th1) cells was detected in the spleen (10.7% vs. 2.17%; *P* < 0.05; Figure 3(b)).

IFN-*γ* activates macrophages and causes their aggregation around Th1 cells, eventually leading to the formation of mature macrophages that are potent killers. These mature macrophages in turn activate more naïve CD4+ cells to differentiate into Th1 cells, thereby forming a positive feedback loop.

As Th1 cells and type-1 cytokines such as IFN-r play a key role in allo-reaction, to further support our hypothesis, we determined the expression of IFN-*γ* in the culture supernatants of splenocytes via culturing and analyzing the cells by ELISA. We found markedly reduced IFN-*γ* levels in the culture supernatants of splenocytes in the rocaglamide-treated group compared with the control group (*P* < 0.001; Figure 3(c)). Particularly, we observed a significant decrease in the serum IFN-*γ* levels in the treatment group (*P* < 0.01; Figure 3(c)), thus indicating that rocaglamide protects the grafts by suppressing the CD4+ IFN-*γ*+ (Th1) cells and preventing the secretion of IFN-*γ* in the peripheral blood.

In addition, we observed lesser lymphocytic infiltration and changes in the number of myocardial cells previously. Hence, we determined the expression of graft rejection-related genes by using mRNA extracted from cardiac allografts and performing qRT-PCR. As shown in Figure 3(d), the levels of IFN-*γ* were suppressed in the treatment group (*P* < 0.05). Meanwhile, immunohistochemical staining for IFN-*γ* was performed in the grafts. IFN-*γ*+ cells showed that the extent of IFN-*γ* infiltration in the treatment group was lower than that in the control group (Figure 3(e)), thus indicating that rocaglamide decreased the accumulation and aggregation of IFN-*γ*.

### 3.4. Rocaglamide-Treated Prolong Allograft Survival Is Associated with Suppressing Th17 Cells, Cytokine Expression of Th17 T Cells, and IL-17 Infiltration

T helper 17 cells (Th17) secreting interleukin-17 (IL-17) are a subset of proinflammatory T helper cells [26]. Guglani and Khader reported that solid graft rejection was related to the number of Th17 cells in multiple transplant models [27]. To further confirm our hypothesis, we examined the number of Th17 cells in the allografts by flow cytometry. The rocaglamide-treated group showed a significant decrease in Th17 cells (1.89%) in the lymph nodes compared with the control group (6.88%; *P* < 0.01, Figure 4(a)). Moreover, the number of CD4+ IL-17+ (Th17) cells was reduced to 3.87% in the spleen compared with that in the control group (6.21%; *P* < 0.01, Figure 4(b)).

Th17 cells differentiate because naïve T cells are induced by TGF-*β*, IL-6, and IL-21 [28]. A previous study suggested that the Th17 subset is the cause of IL-17-dependent graft rejection [1]. Consistent with the findings of Deng et al. and Mandy et al. [1, 29], we found that IL-17 produced by Th17 cells may play a key role in allograft rejection and its secretion was prevented by rocaglamide. To further confirm this finding, we used an ELISA kit to determine the IL-17 levels in culture supernatants. The rocaglamide-treated group exhibited a decrease in IL-17 levels compared with the control group (*P* < 0.05, Figure 4(c)). We observed no statistical significance in serum IL-17 levels between the two groups, but the treatment group showed a slight decrease in IL-17 levels (Figure 4(c)). Recently, retinoid acid-related orphan receptor gamma t (ROR-*γ*t) has been shown to play an important role in the differentiation of Th17 cells, including the secretion of IL-17 [30, 31]. To determine the role of ROR-*γ*t, we determined the gene expression of ROR-*γ*t in the grafts. Although there was no statistical difference, ROR-*γ*t gene expression was downregulated in the rocaglamide-treated group (Figure 4(d)), which may be associated with the decrease in Th17 cells and IL-17 levels.

Furthermore, to evaluate the contribution of Th17 cells within the acute rejection infiltrates, we performed immunohistochemical analysis, which showed that the extent of IL-17 infiltration was markedly reduced in the rocaglamide-treated group (Figure 4(e)).

### 3.5. Rocaglamide Decreases the Memory T Cells but No Effect on Tregs

Memory T cells, including CD4+ and CD8+ subsets, play a crucial role in accelerated rejection [32]. Moreover, several studies have suggested that memory T cells also play a key role in accelerated rejection [33, 34]. To determine whether rocaglamide administration affected the production of effector memory T cells (CD40highCD62low), we analyzed the T lymphocytes obtained from the spleen of recipient mice by flow cytometry.

Interestingly, we found that the CD4+ memory T cells (CD40highCD62low) in the rocaglamide group were suppressed compared with the control group (17.0% vs. 24.2%, *P* < 0.05, Figure 5(a)). In addition, as several studies indicated that the CD4+ Foxp3+ T cells (Tregs) regulate immune response and induce tolerance, we determined the expression of Tregs but no statistically significant difference was observed (Figure 5(b)).

### 3.6. Rocaglamide Treatment Changes Cytokine Expression of Allograft Recipients

In our previous study, we demonstrated that rocaglamide suppresses the expression of IFN-*γ* and IL-17. Interleukin-6 (IL-6) is also a key factor involved in the differentiation of Th17 formation, and hence, we detected its levels in the culture supernatants of splenocytes and serum samples by ELISA. The IL-6 levels in the culture supernatants of the treatment group were significantly lower compared with that in the control group (*P* < 0.001, Figure 6(a)). Moreover, their levels were decreased in the serum (*P* < 0.001, Figure 6(a)). Interleukin-4 (IL-4) is associated with Th2 responses. However, we found no statistical difference in the IL-4 levels between the two groups (Figure 6(b)). We also did not observe statistically significant differences in the interleukin-10 (IL-10) levels in the serum and culture supernatants (Figure 6(c)). Transforming growth factor-beta (TGF-*β*) is produced by regulatory T cells (Tregs) and suppresses immune responses. Moreover, TGF-*β* contributes to the formation of Th17 cells [35]. We found no significant differences between the two groups but found a decrease in TGF-*β* levels in the rocaglamide-treated group, both in the culture supernatants and serum (Figure 6(d)), indicating that low expression of TGF-*β* is good for suppressing Th17 cells but has no positive effect on the formation of Tregs.

These findings may indicate that rocaglamide suppresses the differentiation of naïve CD4+ cells into Th1 cells and Th17 cells and inhibits the secretion of cytokines such as IFN-*γ*, IL-6, and IL-17.

### 3.7. Rocaglamide Affects the Immune Response Ability of T Cells to the Same Identical Gene Tissues

Next, we determined the effect of rocaglamide on the spleen of recipients. After posttransplantation day 7, splenic T cells were isolated for MLR assays, and spleen cells from BALB/c mice (no proliferation ability was noticed after treatment with mitomycin C) were used as the antigen. Our results showed that the proliferation of T lymphocytes in the treatment group was significantly inhibited compared with that in the control group (*P* < 0.001) (Figure 6(e)).

### 3.8. Rocaglamide Suppresses the Nuclear Expression of NF-AT but Not of NF-*κ*B

The inducible transcription factors NF-AT and NF-*κ*B, which are ubiquitous, affect the activation of many inflammatory cytokine genes. Furthermore, according to the previous data, rocaglamide treatment inhibited the proliferation of Th1 and Th17 cells. We hypothesized that rocaglamide might inhibit NF-ATc1, AP-1, and NF-*κ*B expression, which might reversely regulate mTOR expression and negatively regulate the immune response. To determine whether rocaglamide affects the nuclear expression levels of NF-AT and the NF-*κ*B subunit p65 in activated T cells, we extracted nuclear proteins from Jurkat T cells that were stimulated by PMA/ionomycin for 2 h with or without rocaglamide. The nuclear levels of NF-AT caused dose-dependent downregulation of T cell activation (Figure 6(f)). However, at this concentration, rocaglamide had no inhibitory effect on NF-*κ*B activity (Figure 6(g)).

### 3.9. Rocaglamide Inhibits NF-AT via Activation of the MAPKs, JNK, and p38

There are two different ways to activate the NF-AT family of proteins: one is activation via the calcium/calmodulin-dependent phosphatase calcineurin, which phosphorylates and promotes nuclear translocation of NF-AT. However, a recent study [36] suggested that rocaglamide has no direct inhibitory effect on calcineurin activity. Previous studies indicated that the cellular MAPKs, JNK, and p38 can also regulate the nuclear expression of NF-AT. Therefore, to determine the mechanism of the rocaglamide-mediated inhibition of NF-AT activity, we determined the effect of rocaglamide on p38 and pJNK expression. Jurkat T cells were treated with PMA/ionomycin for 2 h with or without rocaglamide. We found that rocaglamide promoted the phosphorylation of p38 without stimulation and enhanced the phosphorylation of pJNK and p38 in the stimulatory environment (Figure 6(h); Figures 7(a) and 7(b)).

To demonstrate whether the activation of MAPKs by rocaglamide induced the reduction in NF-AT activity, Jurkat T cells were treated under the same conditions described previously. The p38 kinase and JNK inhibitors “SB203580” and “SP600125” were, respectively, used depending on the different groups. Group A was administered with normal treatment, group B was treated with the p38 kinase inhibitor (SB 203580), and group C was treated with the JNK inhibitor (SP600125). Data analysis showed that these inhibitors significantly inhibited the rocaglamide-enhanced phosphorylation of p38 (Figures 8(a) and 8(b), the first row). The phosphorylation of pJNK was also inhibited by these inhibitors (Figures 8(a) and 8(c), the second row; Figure 7(b)); however, rocaglamide did not promote the phosphorylation of ERK, and there were no significant differences in ERK activities in these three groups (Figures 8(a), 8(b), and 8(c), the third row). The inhibitors inhibited p38 and JNK phosphorylation and prevented the rocaglamide-induced decrease in NF-AT levels (Figures 8(a), 8(b), and 8(c), the fourth row). At the same time, as a control, we examined the nuclear levels of the NF-*κ*B subunit p65 and found no differences in the same experiments (Figures 8(a), 8(b) and 8(c), the fifth row). Therefore, the inhibition of p38 and JNK phosphorylation prevented a rocaglamide-mediated decrease in NF-AT nuclear export. These results demonstrated that rocaglamide-mediated inhibition of NF-AT activity is correlated with the upregulation of JNK/p38.

## 4. Discussion

The production, differentiation, and activation of T cells play a key role in the immune responses that mediate acute rejection by secreting different types of cytokines. Oxidative stress responses along with the inflammatory cell infiltration of allografts result in the production of cytokines and proinflammatory adhesion molecules, which are the main factors causing vasculopathy and organ injury [37]. First, IFN-*γ* is secreted by Th1 cells at the start of immunoreaction and oxidative stress damage. Second, IFN-*γ* is not only an important activator of macrophages and inducer of class II major histocompatibility complex molecule expression but also an inducer of more undifferentiated naïve CD4+ cells (Th0 cells) that differentiate into Th1 cells [38, 39]. Therefore, a positive feedback loop is formed. Some studies have demonstrated that rocaglamide blocks inducible NF-*κ*B DNA-binding activity and IkBa degradation, which in turn downregulates NF-*κ*B gene expression in T lymphocytes [12].

To the best of our knowledge, this is the first study to report that during transplantation, rocaglamide prolongs allograft survival by reducing the number of CD4+ IFN-*γ*+ (Th1) cells by not only decreasing the number of Th1 cells in the lymph nodes but also in the spleen. Th1-type cytokines such as IFN-*γ* and TNF-*α* stimulate cell-mediated immunoreaction, which causes cytokine production and inflammatory cell aggregation, resulting in more oxidative stress damage and vasculopathy. Thus, the expression of these cytokines is harmful to grafts and causes their rejection. Some recent studies showed that rocaglamide suppresses the secretion of IFN-*γ* and IL-4 in vitro [11, 40]. Interestingly, we first demonstrated that rocaglamide has a suppressive effect on the expression of IFN-*γ* in culture supernatants, peripheral blood samples, and allografts. By analyzing the MLR, we assumed that rocaglamide suppressed the proliferation of T lymphocytes, and eventually, low levels of IFN-*γ* led to lower levels of cytotoxic mediators, lower activation of T cells, and lower differentiation of naïve CD4+ T cells into the Th1 cells. This sequence of events thus formed another positive feedback loop.

Moreover, Becker et al. reported that rocaglamide promotes mitochondria-mediated apoptosis in leukemia cells [11], which is associated with CD95/CD95L-mediated apoptosis in T cells. And CD95L is a known NF-AT target gene [41]. A previous study also showed that mTOR directly affects NF-AT-P, and mTOR signaling plays a key regulatory role in the differentiation and activation of Th1 cells [42]. According to our data, rocaglamide downregulated the expression of NF-ATc1, which is correlated with the inhibition of Th1 cell differentiation.

Baumann et al. and Goriely also reported that rocaglamide could inhibit IL-4 production in Jurkat T cells [12, 36]. However, we found no statistical significance of IL-4 levels between the two groups. Another study suggested that the Th17 subset is crucial for rejection and myocardial injury [27]. Th17 cells generate proinflammatory cytokines such as IL-17A, IL-21, and IL-22 [43]. Sica et al. also demonstrated that decreased Th17 cells promote graft survival by reducing the production of interleukin-17 (IL-17) [44]. Several inducible transcription factors such as AP-1 (Fos/Jun) and NF-AT regulate the secretion of IL-4, IFN-*γ*, and TNF-*α* [45, 46]. We also first reported that rocaglamide could inhibit the differentiation of CD4+ cells into Th17 cells in our cardiac transplantation model. Furthermore, a reduction in IL-17 levels was observed in culture supernatants, serum samples, and allografts. Meanwhile, as shown previously [31], we found that the expression of IL-6, which is associated with proliferation of Th17 cells, was decreased significantly.

Allograft rejection is promoted, and allograft tolerance is prevented via memory T cells in hosts' immune repertoire [34]. Consistent with the findings of previous studies, Pepper et al. reported that the inhibition of CD27/70 reduced the generation of memory T cells [47]. Naïve CD4+ T cells sustainably proliferate and differentiate into different types of helper T cell lineages, including Th1, Th2, and Th17, when exposed to an antigen. Th1 memory cells are produced in vivo after exposure to infection and are differentiated from T-bet and IFN-c-expressing Th1 effector cells [48]. Th1 memory cells showed minimal (or possibly delayed) reexpression of CD62L and CCR7, indicating that these cells are Th1 effector memory cells [47]. Pepper et al. also found that 60% of T-bet+ CXCR5- Th1 memory cells produced IFN-*γ* and IL-2 [47]. A few recent studies showed that IFN-*γ*, IL-17, and IL-4 affect the differentiation and functions of helper T cells of different lineages to some extent. However, the mechanisms by which helper T cells and cytokines promote memory T cells are still unclear. Interestingly, consistent with previous results describing the inhibition of Th1 cells and the expression of IFN-*γ* and IL-17, we found that rocaglamide suppressed the production of effector memory T cells (CD40highCD62low) in the lymph nodes.

Regulatory T cells are usually required for the prolongation and tolerance of a transplant; however, we found that rocaglamide did not affect CD4+ Foxp3+ T cells. Growth factor-beta (TGF-*β*) and IL-10, which inhibit helper T cells, also showed no statistical significance.

In summary, our present findings showed that rocaglamide therapy led to a significant prolongation of allograft survival, which was associated with significantly reduced Th1 cells and IFN-*γ*, low levels of IFN-*γ* that led to lower cytotoxic mediators, lower activation of T cells, and lower differentiation of naïve CD4+ T cells into Th1 cells. Furthermore, this is the first study to report that rocaglamide suppressed the differentiation of naïve CD4+ T cells into Th17 cells, thereby also inducing the marked decrease in IL-17 levels, which might be associated with the inhibition of IL-6. We also found that the phosphorylation of JNK and p38, which are key regulators of NF-AT and indispensable for activating the transcription of cytokine genes, was enhanced by rocaglamide treatment. However, the inhibitory role was nullified when the p38 kinase (SB203580) and JNK inhibitors (SP600125) were used. Overactivation of p38 and JNK may lead to rocaglamide-mediated inhibition of NF-AT activity.

These results indicated that the suppression of Th1 cell proliferation, activation, and differentiation, which might be associated with the expression of NF-AT, was inhibited. Although the mechanisms of the effect of rocaglamide on antigen-presenting cells in oxidative stress injury and transplantation immunity need to be determined, our findings may facilitate the development of a new therapy for IFN-*γ*- and IL-17-mediated rejection and inflammation.

## 5. Conclusion

We found that rocaglamide could be potentially used for preventing cell-mediated acute rejection and alleviating oxidative stress because it prevents T helper cell differentiation and T cell-mediated cytokine secretion. We also found that the suppressive effect of rocaglamide on T helper cell proliferation, activation, and differentiation could be associated with the inhibition of NF-AT expression.

Our results clearly demonstrate a novel immunoregulatory property of rocaglamide, wherein it regulates oxidative stress response and reduces inflammatory cell infiltration and organ injury. Our findings could be useful for surgeons performing organ transplantation and immunologists studying transplantation immunity and inflammatory factors.

## Figures and Tables

**Figure 1:** Administration of rocaglamide further prolongs graft survival. (a, b) Survival of the graft in cardiac transplantation (Kaplan–Meier plot). Recipients were treated with rocaglamide, and the heart grafts survived for 25 days (median survival). Rocaglamide treatment revealed significantly reduced inflammatory cell infiltration and protected the myocardial architecture. Photographs shown in this figure are representative of 3 animals in each group (a, b: 100x, 200x). (c) The International Society of Heart and Lung Transplantation (ISHLT) scores of the hearts, with each spot representing the score from each slice. The horizontal line represents the mean for each group (*n* = 6 in each group; ^∗^*P* < 0.05, ^∗∗^*P* < 0.01, and ^∗∗∗^*P* < 0.001).

**Figure 2:** Administration of rocaglamide inhibits the T cell activation in allograft recipients. (a) Freshly isolated lymphocytes and splenocytes were stained for CD3 and assayed for the incidence of CD3+ cells in the transplantation recipients. Data are presented for a representative experiment of at least three experiments (*n* = 3; ^∗^*P* < 0.05, ^∗∗^*P* < 0.01, and ^∗∗∗^*P* < 0.001). (b, c) Analyzing the proportion of CD11b+ and CD11c+ antigen-presenting cells in the spleen. (d, e) Proportion of CD11b+ CD80+ cells and CD11c+ CD86+ cells in the spleen. (f, g, and h). Freshly isolated lymphocytes and splenocytes were stained for CD134 (OX40), CD69, and CD44 expression and assayed for the evidence of T cell activation in the transplantation recipients (blue represents the fluorescence intensity of the treatment group, and the red represents the control group).

**Figure 3:** Rocaglamide administration decreases Th1 cells, cytokine expression of Th1 T cells, and accumulation of IFN-*γ* in allograft recipients. (a) Analyzing the proportion of CD4+ IFN-*γ*+ cells (Th1) in the lymph nodes using fluorochrome-conjugated-specific antibodies detected by flow cytometry. Data are presented for a representative experiment of at least three experiments (*n* = 3; ^∗^*P* < 0.05, ^∗∗^*P* < 0.01, and ^∗∗∗^*P* < 0.001). (b) Proportion of CD4+ IFN-*γ*+ cells (Th1) in splenic lymphocytes. (c) Expression of IFN-*γ* in the peripheral blood and culture supernatants detected by ELISA kits. (d) mRNA extracted from cardiac grafts and analyzed by qRT-PCR. The rocaglamide-treated group showed decreased IFN-*γ* in allografts when compared with the control group (^∗^*P* < 0.05). (e) Rocaglamide decreases the accumulation and aggregation of IFN-*γ* (a: 100x, 200x) in cardiac grafts. Immunohistochemical staining was performed, and the data showed the infiltration of IFN-*γ* was diminished in the rocagalmide-treated group.

**Figure 4:** Rocaglamide-treated prolonged allograft survival is associated with suppressing Th17 cells, cytokine expression of Th17 T cells, and IL-17 infiltration. (a) Flow cytometric analysis rocaglamide-treated prolonged allograft survival is associated with suppressing Th17 cells in lymph nodes (*n* = 3, ^∗^*P* < 0.05, ^∗∗^*P* < 0.01, and ^∗∗∗^*P* < 0.001). (b) Th17 cells in splenic lymphocytes were also suppressed. (c). Expressions of IL-17 in the peripheral blood and culture supernatants were tested by ELISA kits (*n* = 3, ^∗^*P* < 0.05, ^∗∗^*P* < 0.01, and ^∗∗∗^*P* < 0.001). (d) mRNA was extracted from cardiac grafts and analyzed by qRT-PCR. The rocaglamide-treated group showed decreased ROR-*γ*t in allografts when compared with the control group. (e) Rocaglamide decreases the accumulation and aggregation of IL-17 (b: 100x, 200x) in cardiac grafts. Immunohistochemical staining was performed, and the data showed that the infiltration of IL-17 was diminished in the rocagalmide-treated group.

**Figure 5:** Rocaglamide decreases the memory of T cells, but no effect was noted on Treg. (a) Flow cytometric analysis of memory T cells (CD40highCD62low) considers the proportion of lymphocytes (*n* = 3; ^∗^*P* < 0.05, ^∗∗^*P* < 0.01, and ^∗∗∗^*P* < 0.001). (b) Flow cytometric analysis of CD4+ Foxp3+ regulatory T cells (Tregs).

**Figure 6:** Rocaglamide treatment changes the cytokine expression of allograft recipients, affects the immune response ability of T cells to the same identical gene tissues, and suppresses the nuclear expression of NF-AT, but not that of BF-Kb. (a–d) The levels of IL-6 (a), IL-4 (b), IL-10 (c), and TGF-*β* (d) in the serum and supernatants curve from MLR were detected by using commercially available ELISA kits. Each reaction was conducted in triplicate (^∗^*P* < 0.05, ^∗∗^*P* < 0.01, and ^∗∗∗^*P* < 0.001). (e) To investigate the effectiveness of rocagalmide on the proliferation of T cells, both in the spleen and lymph nodes, and we performed mixed lymphocyte reaction assays. Data from three separate wells were dedicated to each responder-stimulator, and each experiment was repeated thrice (*n* = 3; ^∗^*P* < 0.05, ^∗∗^*P* < 0.01, and ^∗∗∗^*P* < 0.001). (f) T cell activation induced by the nuclear expression of NF-AT was downregulated. Jurkat T cells were stimulated with PMA and ionomycin for 2 h with or without rocaglamides (added 1 h before stimulation). Nuclear proteins were extracted and immunoblotted with mAb against NFATc1. (g) The nuclear proteins were immunoblotted with Abs to p65. (h) Rocaglamides activate MAPKs, p38, and JNK. Jurkat T cells were stimulated with PMA and ionomycin for 2 h in the absence or presence of various concentrations of rocaglamides (added 1 h before stimulation). Total cell lysates were immunoblotted with Abs against phosphorylated p38 (p-p38) and phosphorylated JNK.

**Figure 7:** Rocaglamide inhibits Th1/Th17 cell differentiation and prolonged graft survival through NF-AT pathway downregulation. (a) Recipients were treated with PBS (*n* = 6) and rocaglamide (*n* = 8) for survival studies. Heart grafts were monitored until they stopped beating. Grafts were performed, and recipients were sacrificed on day 7 for histological, MLR, ELISA, PCR, and flow cytometric analysis. RNA was extracted from the grafts of recipient mice. (b) Rocaglamides inhibit NF-AT via the activation of MAPKs, and rocaglamide can enhance the phosphorylation of pJNK and p38 in the simulation environment. Rocaglamide suppresses the nuclear expression of NF-AT in activated T cells. Rocaglamide suppresses the activation of T cells and reduces naive CD4+ T cell differentiation into Th1/Th17 cells. Moreover, it decreases the secretion of IFN-*γ* and IL-17; thus, in turn, low-level expression of IFN-*γ* leads to lower cytotoxic mediators, lower activation of T cells, and lower differentiation of naive CD4+ T cells into the Th1 cells. A feedback loop then begins. However, the inhibition of p38 and JNK phosphorylation prevented rocaglamide-mediated decrease of NF-AT nuclear export.

**Figure 8:** Rocaglamide inhibits NF-AT via activation of the MAPKs, JNK, and p38. Jurkat T cells were treated with same condition described previously, and p38 kinase and JNK inhibitors (SB 203580 and SP 600125) were used, respectively, depending on the different group. Group A was normal treated, group B was treated with p38 kinase inhibitor (SB 203580), and group C was treated with JNK inhibitors (SP600125).

## Data Availability

Previously reported data were used to support this study and are at available relevant places within the text as references. The new data used to support the findings of this study may be released upon application to the Institute of Organ Transplantation, Tongji Hospital, Tongji Medical College, Huazhong University of Science and Technology; Key Laboratory of Organ Transplantation, Ministry of Education; NHC Key Laboratory of Organ Transplantation; Key Laboratory of Organ Transplantation, Chinese Academy of Medical Sciences, Wuhan, China. 430030, Zhishui Chen, Wuhan, China. Tel. +86 27 83665203 can be contacted at the corresponding author upon request.

## Supplementary Materials

Supplementary 1 Supplemental Figure 1: rocaglamide decreased the expression of AP-1. Rocaglamides activate MAPKs, p38, and JNK. Jurkat T cells were stimulated with PMA and ionomycin for 2 h in the absence or the presence of various concentrations of rocaglamides (added 1 h before stimulation). Total cell lysates were immunoblotted with Abs against c-Jun.

Supplementary 2 Supplemental Figure 2: rocaglamide had no effect on apoptosis in the activated condition flow cytometric analysis rocaglamide-treated cells. We measured apoptosis levels with and without rocaglamide in activated conditions. As shown in the figure below, we found that rocaglamide had no effect on apoptosis in the activated condition. This phenomenon has been discussed in our article.

Supplementary 3 Supplemental Figure 3: rocaglamide had no effect on B cells in the recipients. A. Analyzing the proportion of CD19+ using fluorochrome-conjugated-specific antibodies detected by flow cytometry. Data are given one representative experiment of at least three experiments (*n* = 3; ^∗^*P* < 0.05, ^∗∗^*P* < 0.01, and ^∗∗∗^*P* < 0.001). B. Serum alloantibody measurement, IgG, and IgM antibodies were analyzed by ELISA. We found that rocaglamide therapy could not reduce the number of CD19+ B cells (A). We found that there was slightly decrease tendency on IgG of recipients treated with rocaglamide, but there was no statistical significance; meanwhile, there were no differences on IgM also (B).
